The article "Correlation between Palpitations below the Heart in Traditional Chinese Medicine and Autonomic Nerve Function Based on Heart Rate Variability: A Case-Control Study" was published in 2021. Journal: Evid Based Complement Alternat Med.

# Correlation between Palpitations below the Heart in Traditional Chinese Medicine and Autonomic Nerve Function Based on Heart Rate Variability: A Case-Control Study

**DOI:** 10.1155/2021/1945488

**Published:** 2021-10-31

**Authors:** Chengcheng Song, Kelong Chen, Ziqian Wu, Wei Liu, Ling Chen, Wenzong Zhu

**Affiliations:** Department of Neurology, Wenzhou Municipal Hospital of Traditional Chinese Medicine, Wenzhou, China

## Abstract

**Objective:**

To explore the autonomic nerve rhythm and the correlation between palpitations below the heart (PBTH) and autonomic nerve function in patients with PBTH based on heart rate variability (HRV).

**Methods:**

The outpatients or ward patients of Wenzhou Hospital of Traditional Chinese Medicine were collected and divided into two groups: the PBTH group and the normal group. The HRV of each group was detected. Single-factor statistical methods, Spearman correlation analysis, and logistic regression were used to describe and analyze the rhythm and characteristics of autonomic nerves in patients with PBTH and the correlation between PBTH and autonomic nerve function.

**Results:**

(1) In the comparison of HRV in different time periods in the same group, the SDNN, RMSSD, pNN50, TP, and HF in the PBTH group at night were significantly higher than those in the daytime (*P* < 0.01), while the LF/HF ratio was significantly lower than that in the daytime (*P* < 0.01). (2) In the comparison of HRV between the two groups in the same time period, the RMSSD and pNN50 of the PBTH group during the daytime period were significantly higher than those of the normal control group (*P* < 0.05), and the LF/HF was significantly lower than that of the normal group (*P* < 0.05). (3) In the Spearman correlation analysis, PBTH was significantly correlated with RMSSD, pNN50, and LF/HF ratio in the daytime period, with correlation coefficients of 0.424, 0.462, and −0.524, respectively (*P* < 0.05). (4) Logistic regression analysis showed that the decrease of LF/HF ratio during the daytime period was an independent risk factor for PBTH in TCM (OR = 0.474, 95% CI: 0.230–0.977, *P* < 0.05).

**Conclusions:**

The changes in parasympathetic nerve function in patients with PBTH have a circadian rhythm, which is characterized by increased activity during the nighttime. At the same time, the autonomic nerve activity of people with PBTH during the daytime is unbalanced, and the decrease of LF/HF ratio during the day is an independent high risk factor for PBTH.

## 1. Introduction

Palpitations below the heart (PBTH) is a common clinical syndrome characterized by “conscious subcardiac epigastric beating,” “throbbing at the lower part of the heart,” and “palpitation rhythm consistent with the pulse and obvious pulse in the heart area,” accounting for about 14% of all clinical abdominal syndromes [1], which seriously affect the quality of life of patients. Even though our team has initially established the corresponding standard of PBTH in TCM based on the Delphi method in the early stages [2], there are few further objective studies concerning PBTH all over the world, and the research on its internal related factors and mechanism has not been carried out yet, so there is no obvious progress in the treatment of it in medicine. In other words, the discussion of the underlying factors and mechanism of PBTH will be the focus of the next research and has far-reaching significance.

The article "Correlation between Palpitations below the Heart in Traditional Chinese Medicine and Autonomic Nerve Function Based on Heart Rate Variability: A Case-Control Study" was published in 2021. Journal: Evid Based Complement Alternat Med.

Based on the previous analysis of the ancient literature, clinical symptoms, similar research, and pharmacology of effective drugs, we preliminarily believe that there may be a certain relationship between PBTH and autonomic nerve function [3]. The related diseases and syndromes of PBTH have been recorded in *Treatise on Febrile and Miscellaneous Diseases* in detail. The records of clinical symptoms include “excessive sweating,” “dizziness and desire to fall,” “alternating spells of fever and chills,” “inhibited urination,” and “cold limbs,” which coincides with the clinical manifestations of the imbalance of autonomic nervous function leading to the regulation of internal organs, such as the digestive tract, cardiovascular, and endocrine dysfunction [4]. In addition, the ancient book of TCM, *A Survey of Abdominal Syndrome*, often describes the abdominal syndrome of PBTH as “Abdominal Syndrome of Guizhi Decoction” and “Syndrome of Guizhi Gancao Decoction,” which indicates the exact curative effect of Guizhi decoction on palpitations [5]. At present, many pharmacological studies have confirmed that Guizhi decoction plays a therapeutic role by regulating autonomic nerve balance and repairing sympathetic and vagus nerve function [6], which is instructive for the further study of the relationship between PBTH and autonomic nerve function. In further sorting out the research on PBTH, it is found that although many physicians believe that PBTH is related to the pulsation of the abdominal aorta, there is still a lack of further research to explain the relationship [7]. Similar studies of PBTH in other parts, however, indicate that PBTH is more likely to be related to autonomic nervous imbalance [8]. Therefore, we put forward the scientific hypothesis that PBTH is closely related to autonomic nerve function and designed objective scientific research to reveal it.

Heart rate variability (HRV), as a well-known quantitative index of autonomic nervous function, has the advantages of objectivity and sensitivity compared with other detection methods, such as postural blood pressure test, skin sympathetic response, and Wagner motion response index, which is suitable for a wide range of applications [9, 10]. At present, the methods to evaluate HRV include time domain, frequency domain, and nonlinear analysis [11]. Nonlinear analysis is still in the research stage and is not used as a routine analysis method to evaluate HRV. Time domain analysis and frequency domain analysis have clear significance and mature theory, which have been widely used in the study of TCM constitution and syndrome types [12]. The time domain indexes mainly include SDNN, RMSSD, SDANN, and pNN50. Among them, SDNN reflects the regulation ability of the total autonomic nerve; RMSSD measures the activity of the vagus nerve; SDANN reflects the activity intensity of the sympathetic nerve; and pNN50 is the percentage of the total number of beats with the difference between the two adjacent sinus R-R intervals greater than 50 ms. When the heart rate is in sinus rhythm, pNN50 has the same meaning as RMSSD, showing the activity of the vagus nerve [13]. The indexes of the frequency domain analysis method are mainly divided into total power (TP), low-frequency (LF) band, high-frequency (HF) band, and the ratio of low frequency to high frequency (LF/HF). Among them, TP represents the overall regulation ability of the autonomic nerve. The value of LF is affected by the function of the sympathetic and parasympathetic nerves, but it is mainly regulated by the sympathetic nerve. Some studies have also proposed that the change of LF represents the rhythm change of the sympathetic nerve, and LF oscillation is a fundamental property of central autonomic outflow [14, 15]. In addition, LF oscillation is also affected by baroreflex function, which is disturbed by rhythmically influencing the aortal nerve and the carotid sinuses [16]. HF reflects the activity of the parasympathetic nerve, and LF/HF is usually used to indicate the balance between the sympathetic nerve and the parasympathetic nerve.

The article "Correlation between Palpitations below the Heart in Traditional Chinese Medicine and Autonomic Nerve Function Based on Heart Rate Variability: A Case-Control Study" was published in 2021. Journal: Evid Based Complement Alternat Med.

To sum up, in this study, we try to explore the correlation between PBTH and the autonomic nerve by HRV analysis, hoping to provide evidence-based study for clinical diagnosis and treatment of PBTH and play a positive role in promoting further scientific research of PBTH.

## 2. Materials and Methods

### 2.1. Subjects

A total of 24 cases were included in this study, including 16 cases in the PBTH group and 8 cases in the normal group, all from the outpatients and ward patients of Wenzhou Hospital of Traditional Chinese Medicine. The diagnostic criteria for PBTH come from the expert consensus based on the Delphi expert consultation method [2]. The primary diagnosis of PBTH included “conscious subcardiac epigastric beating,” “throbbing at the lower part of the heart,” and “palpitations rhythm consistent with the pulse and obvious pulsation in the heart area.” The secondary diagnosis is “palpitations obvious after nervous tension, fatigue, drinking water, or changing body position.” The inclusion criteria were as follows: those who met the abovementioned diagnostic criteria for palpitations, aged between 20 and 30 years, with sinus rhythm on ECG and no previous heart disease, and who were familiar with and signed the informed consent. The exclusion criteria were as follows: patients with previous cardiac surgery or pacemaker implantation; patients with hypertension, diabetes, mental illness, malignant tumors, and severe hepatic and renal insufficiency; pregnant or lactating women; patients who had taken drugs affecting heart rate within 3 months, including beta-blockers, sodium, or calcium channel blockers, and cardiotonic drugs; and those who were currently participating in clinical trials of other drugs. This comparative open study was conducted at Wenzhou Hospital of Traditional Chinese Medicine, and all subjects completed it successfully.

### 2.2. Ethical Approval

This study was approved by the Ethics Committee of Wenzhou Hospital of Traditional Chinese Medicine (approval number: WTCM-KT-2020070). Each subject was informed of the purpose and risk of the study and signed an informed consent form before the study.

### 2.3. Data Collection

The basic information of each subject was inquired, collected, and recorded by the research members, including the name, gender, age, height, weight, body mass index, personal contact information, address, medical history, medication, and vital signs of the subjects. The time domain and frequency domain analysis methods of linear analysis method in HRV were used in this study. The time domain indexes were expressed in ms, including SDANN, the standard deviation of the mean value of every 5 min interval, reflecting sympathetic nerve tension; SDNN, the standard deviation of normal sinus interval, reflecting the overall HRV; RMSSD, the root mean square value of the difference between adjacent intervals, reflecting vagal nerve tension; pNN50, the percentage of the total number of beats whose interval difference between two adjacent sinus beats is more than 50 ms. When the heart rate is in sinus rhythm, pNN50 has the same meaning as RMSSD; both of them show the activity of the vagus nerve. The frequency domain indexes were expressed in ms^2^, including total power (TP), reflecting the overall autonomic nervous function state; low-frequency (LF) power, reflecting the composite regulation of the sympathetic and vagal nervous system, which mainly reflects sympathetic tension; high-frequency (HF) power, reflecting the function of the vagus nerve regulation; and the ratio of low-frequency power to high-frequency power (LF/HF), reflecting the balance between the sympathetic nerve and vagus nerve.

The article "Correlation between Palpitations below the Heart in Traditional Chinese Medicine and Autonomic Nerve Function Based on Heart Rate Variability: A Case-Control Study" was published in 2021. Journal: Evid Based Complement Alternat Med.

### 2.4. Holter Protocols

The experimental instrument used for monitoring and recording ECG in this study is the SE-2003 24-hour Holter with 3 channels and 7 electrodes produced by China Shenzhen Libang Precision Instrument Co., Ltd. The HRV index is calculated and generated by the analysis software that comes with the Holter machine. To ensure the accuracy of monitoring data, the Holter instrument needs to be corrected before wearing. Then, according to the connection method of 3-channel 7-electrode Holter, the subjects were wearing the instrument. The corresponding lead positions were as follows: (1) lead MV1: the positive pole of lead MV1 is located in the right fourth intercostal space near the right edge of the sternum, which is equivalent to the position of the chest lead V1, and the negative pole is located at the junction of the left clavicle and sternum; (2) lead MV3: the positive pole of lead is located in the middle line of the sixth rib on the left, which is equivalent to the position of the chest lead V3, and the negative pole is located in the middle line of the second rib sternum; (3) lead MV5: the positive pole of the lead is located at the sixth rib of the left axillary front line, which is equivalent to the position of the chest lead V5, and the negative pole is located at the junction of the right clavicle and sternum; and (4) the irrelevant electrode or ground wire is located above the right lowest rib. Holter was worn from 9:00 a.m. to 9:00 a.m. the next day for 24 hours. Among them, 08:00–22:00 is set as day time and 22:00–08:00 is set as nighttime. After 24 hours of normal daily activities, the instrument was removed, and the recorded continuous Holter signals were input into the supporting Holter analysis software for analysis to obtain and record 24-hour HRV information. During the period of wearing the instrument, the subjects were instructed not to engage in strenuous activities.

### 2.5. Statistical Analysis

SPSS 22.0 statistical software was used to establish the database for statistical analysis. The normal data in the measurement data is represented by “mean ± standard deviation,” the nonnormal data is represented by “median (quartile),” and the count data is represented by frequency or constituent ratio. The chi-square test was used to compare the differences of gender distribution among different groups; independent sample *T*-test or nonparametric test was used to compare the age, BMI index, and HRV index between groups (Satterthwaite approximate *t*-test was used for uneven variance in the independent sample *t*-test); Spearman correlation analysis was used to study the relationship between PBTH and related factors; and binary logistic regression was used to analyze the influencing factors of PBTH. All statistical analyses were performed by a two-sided test with the test level set at 0.05.

The article "Correlation between Palpitations below the Heart in Traditional Chinese Medicine and Autonomic Nerve Function Based on Heart Rate Variability: A Case-Control Study" was published in 2021. Journal: Evid Based Complement Alternat Med.

## 3. Results

### 3.1. Demographic Characteristics of Subjects

In this study, a total of 24 cases were included, and 0 case was excluded. There were 16 cases in the PBTH group and 8 cases in the normal group. They were all treated in the outpatient or ward of Wenzhou Traditional Chinese Medicine hospital, including 11 males and 13 females, aged 21–30 years. There were no significant differences in gender, age, height, weight, body mass index, and abdominal circumference between the two groups (*P* > 0.05). The specific baseline characteristics of patients are shown in Table 1.

### 3.2. Comparison of 24-Hour HRV between the Two Groups

The frequency domain and time domain indexes of HRV were compared between the two groups to reflect the difference in autonomic nervous function between the PBTH group and normal control group. The results showed that the SDNN, RMSSD, SDANN, and HF indexes of the PBTH group had a tendency to increase compared with the normal control group, and the TP, LF, and LF/HF indexes had a downward trend compared with the normal group, but the difference between the two groups was not statistically significant (*P* > 0.05). See Table 2 for details.

### 3.3. Comparison of HRV in Different Periods of Day and Night in the Same Group

Compared with the daytime period, the time domain indexes such as SDNN, RMSSD, and pNN50 in the nighttime period of the normal control group were increased. The frequency domain indexes such as TP, HF, and LF were also increased, while the LF/HF ratio was decreased, and the difference was statistically significant (*P* < 0.05). It is suggested that the autonomic nervous activity of normal people is in different regulation state in the daytime and at night. The sympathetic and parasympathetic nerve activities increase in varying degrees at night, especially parasympathetic nerve activity. In addition, the indexes of SDNN, RMSSD, and pNN50 in the nocturnal period of the PBTH group were significantly higher than those in the daytime (*P* < 0.01), the indexes of TP and HF in the frequency domain were also significantly higher (*P* < 0.01), and the LF/HF ratio was significantly lower (*P* < 0.01), but the LF index in the nocturnal period was not significantly higher than that in the daytime (*P* > 0.05). It was suggested that the parasympathetic nerve in the PBTH group has rhythmicity in the circadian period. The activity of the parasympathetic nerve in the PBTH group increases at night, but the regulation of sympathetic nerve activity has little change in different periods. See Table 3 for details.

The article "Correlation between Palpitations below the Heart in Traditional Chinese Medicine and Autonomic Nerve Function Based on Heart Rate Variability: A Case-Control Study" was published in 2021. Journal: Evid Based Complement Alternat Med.

### 3.4. Comparison of HRV between Two Groups in Different Periods of Day and Night

By comparing the indexes of HRV in daytime between the two groups, it was found that the time domain indexes RMSSD and pNN50 of the PBTH group were significantly higher than those of the normal control group (*P* < 0.05) and the frequency domain indexes LF/HF were significantly lower than those of the normal group (*P* < 0.05). Although SDNN, TP, and HF of the PBTH group were higher than those of the normal control group, and LF was lower than that of the normal group, there was no significant difference between the two groups (*P* > 0.05). The results suggested that the balance of sympathetic and parasympathetic nerves in the PBTH group is unbalanced compared with that in the normal group during the daytime, which may be related to the hyperactivity of parasympathetic nerves. Meanwhile, the activity of sympathetic nerves in the PBTH group has a downward trend compared with that in the normal group during this period. There was no significant difference in SDNN, RMSSD, pNN50, TP, LF, HF, and LF/HF between the two groups at night (*P* > 0.05), suggesting that during the night, the autonomic nervous activity of the PBTH group was not significantly changed compared with the normal group. The HRV parameters of the two groups are shown in Table 4.

### 3.5. Spearman Correlation Analysis of PBTH

Spearman correlation analysis was used to study the correlation between PBTH and gender, age, abdominal circumference, body mass index, and HRV. The results showed that PBTH was significantly correlated with RMSSD, pNN50, and LF/HF in the daytime, and the correlation coefficients were 0.424, 0.462, and −0.524 (*P*=0.039,  0.023,  0.009, *P* < 0.05), respectively. There was no statistical significance between PBTH and gender, age, abdominal circumference, body mass index, and other HRV indicators. See Tables 5–7 for details.

### 3.6. Logistic Regression Analysis of Related Factors of PBTH

In this study, PBTH was taken as the dependent variable (0 = no palpitations and 1 = palpitations), the indexes with significant correlation were included in the logistic regression model, and the forward: LR method was used for analysis. Logistic regression analysis showed that the effect of daytime LF/HF on PBTH was statistically significant (*χ*2 = 4.095, *P*=0.043, and *P* < 0.05), while the effects of daytime RMSSD and pNN50 on PBTH were not statistically significant (*P*=0.771, *P*=0.851, and *P* > 0.05). The decrease in daytime LF/HF was a risk factor for PBTH (OR = 0.474, 95% CI: 0.230–0.977). See Table 8 for details.

The article "Correlation between Palpitations below the Heart in Traditional Chinese Medicine and Autonomic Nerve Function Based on Heart Rate Variability: A Case-Control Study" was published in 2021. Journal: Evid Based Complement Alternat Med.

## 4. Discussion

Palpitations below the heart, as a common and enlightening symptom and sign in the clinical work of TCM, has not been paid attention to by doctors of traditional Chinese medicine and Western medicine, which is a pity and needs to be studied and overcome in the future. As an innovative research direction, the early research in this field is not only limited to the lack of recognized diagnostic criteria for PBTH but also limited to the understanding of its internal related factors and mechanisms, which is also the difficulty and focus of the research on PBTH. In recent studies, we have reached an expert consensus on the diagnostic criteria of PBTH based on the Delphi expert consultation method [2] and put forward a scientific hypothesis that there is an intrinsic correlation between PBTH and autonomic nervous function by summarizing the symptoms of PBTH and medication experience [3]. More and more pieces of evidence have confirmed that HRV, as a quantitative objective index of autonomic nervous function, is more accurate and reliable than subjective scale evaluation and has been widely used in autonomic nervous system related research. Therefore, this study analyzes the relationship between PBTH and the autonomic nervous system by investigating the HRV indexes of patients with PBTH, so as to actively promote the research of TCM PBTH.

In the comparison of 24-hour HRV data of the PBTH group and the normal group, the activity of parasympathetic nerve and sympathetic nerve in the PBTH group only showed an upward or downward trend, which was of little significance. However, considering that 24-hour HRV cannot reflect the changes in different periods of day and night and the rhythm regulation of the autonomic nervous system, we analyzed the HRV of the two groups in the daytime and nighttime. Finally, the facts showed that the activity of the autonomic nerve in normal people was in a different regulation state in the daytime and nighttime. The activity of sympathetic and parasympathetic nerves increased to a certain extent in the nighttime, and the increase in parasympathetic nerve activity was more obvious. This result confirmed the circadian rhythm of the parasympathetic nerve in the normal population, which was characterized by increased nighttime activity, which was consistent with the circadian rhythm of the parasympathetic nerve mentioned in existing studies [17]. However, the conclusion of increased sympathetic nerve activity at night in this study is inconsistent with current understanding. The possible explanation was that the effect of the sympathetic nervous system on the increase of HRV was mainly in the early morning period [18], and the nighttime set in this study was exactly 22:00–8: 00, which was easy to cause the measurement at this time to increase false-positive sympathetic nerve activity. On the other hand, although the parasympathetic nerves of people in the PBTH group had rhythmic changes in the circadian period, which was characterized by increased activity during the night period, the adjustment of sympathetic nerve activity in different periods was not obvious. In the comparison of HRV between the two groups at different time periods, the autonomic nerve function activity of the two groups was significantly different in the daytime, which was manifested as the imbalance of autonomic nerve activity and the hyperactivity of the parasympathetic nerve in the PBTH group, but the difference of sympathetic nerve function was not obvious. However, there were no obvious abnormal changes in autonomic nerve activity between the two groups at night. This was partly inconsistent with the scientific hypotheses we put forward based on the rules of symptoms and medications in the early stage of our research. The discrepancy was mainly reflected in the hyperactivity of the parasympathetic nerve rather than the sympathetic nerve in the PBTH group. However, there was no doubt that PBTH was closely related to the imbalance of sympathetic parasympathetic function. One possible explanation is that we neglected that PBTH is the palpitations of a “virtual person” with yang deficiency and phlegm dampness as the disease in the early stage. With more and more studies on the correlation between HRV and TCM syndrome types, many studies have confirmed that in TCM syndrome types, yin syndrome and cold syndrome are mainly manifested as HF increase and LF/HF decrease, that is, the corresponding yang deficiency is more obvious, while the increase of LF is more correlated with yang syndrome and real heat syndrome [19]. At the same time, in the existing research on HRV and TCM physique, yang deficiency physique is also manifested as a decrease in SDANN and LF/HF and an increase in HF. In addition to the decrease in LF/HF, the phlegm-damp constitution also shows a decrease in VLF. Generally speaking, yang deficiency and phlegm dampness are mainly manifested as hyperactivity of the parasympathetic nerve and decrease of sympathetic nerve activity [20, 21], which coincides with the results of this study and is also consistent with the preliminary classification of PBTH syndrome based on the Delphi method. Another possible explanation for this unexpected result is that the medications for PBTH we mentioned earlier do not simply inhibit sympathetic nerves and increase vagus nerve activity, but through the promotion and inhibition of nerve growth factors, they inhibit the hyperproliferation of sympathetic or parasympathetic nerve activity and ultimately play a role in repairing the autonomic nerve function and readjusting the unbalanced sympathetic and vagus nerves to achieve balance.

The article "Correlation between Palpitations below the Heart in Traditional Chinese Medicine and Autonomic Nerve Function Based on Heart Rate Variability: A Case-Control Study" was published in 2021. Journal: Evid Based Complement Alternat Med.

In the further study of related factors of PBTH, we found that PBTH was positively correlated with RMSSD and pNN50 in the daytime (Spearman correlation coefficient 0.424 and 0.462) and negatively correlated with LF/HF in the daytime (Spearman correlation coefficient 0.524). In the subsequent logistic regression analysis, it was found that the decrease of LF/HF in the daytime was a risk factor for PBTH (OR = 0.474, 95% CI: 0.230–0.977). The findings from the current study have important implications for future research. In other words, our results showed that the monitoring of LF/HF ratio during the daytime can be used as an objective predictor of PBTH in the future and also as one of the evaluation indexes of the efficacy of PBTH diagnosis and treatment in the future. At the same time, it may also help to carry out the study of PBTH in people who cannot be clearly diagnosed.

This study is not without limitations. First of all, in order to exclude the influence of age, heart disease, hypertension, diabetes, and other factors on HRV [22–26], this study strictly set the inclusion criteria, in which the age of the population was set at 20–30 to reduce the possibility of suffering from basic diseases affecting the indicators. However, this caused the disadvantages of limited age and small number of cases in the study. In future studies, we need to expand the age stratification and number of cases to further study the autonomic nervous function differences in people with PBTH. In addition, the time periods of this study are 8:00–22:00 and 22:00–8:00, which need to be further subdivided in the later study to further study the rhythm changes of the autonomic nervous system in different periods of PBTH. If necessary, multidisciplinary cooperation of further research, from a multiangle study of PBTH autonomic nerve activity rhythm, will provide an objective theoretical basis for the future of TCM treatment of PBTH. Despite these limitations, results advance knowledge on PBTH. Specifically, this study explored the internal relationship between PBTH and the autonomic nervous system, revealed the changes of the autonomic nervous system rhythm in patients with PBTH, and clarified the high risk factors of PBTH.

The article "Correlation between Palpitations below the Heart in Traditional Chinese Medicine and Autonomic Nerve Function Based on Heart Rate Variability: A Case-Control Study" was published in 2021. Journal: Evid Based Complement Alternat Med.

## 5. Conclusions

In this study, we found that the parasympathetic nerves of people with PBTH have circadian rhythm changes, which are characterized by increased activity during the night, but the circadian rhythm of sympathetic nerve activity is not obvious. At the same time, the autonomic nerve activity of people with PBTH during the daytime was unbalanced, which was manifested by the hyperactivity of their parasympathetic nerves. In addition, this study found that the decrease in the ratio of LF/HF during the day was an independent high risk factor for PBTH, which had certain clinical predictive and diagnostic value for PBTH. It can be seen from the above that patients with palpitations have corresponding characteristics of autonomic neuropathy, which provides a theoretical basis and ideas for future clinical diagnosis and treatment of PBTH and further scientific research.

## Figures and Tables

**Table 1:** Baseline characteristics of the patients.

Group	Gender		Age (years)	Body height (cm)	Body weight (kg)	Body mass index (kg/m^2^)	Abdominal circumference (cm)
	Men	Women					
Palpitations below the heart group	6	10	24.63 ± 2.03	162.94 ± 6.51	51.63 ± 6.46	19.41 ± 1.73	70.75 ± 3.53
Normal group	5	3	23.00 (22.00, 23.75)	168.50 ± 6.65	57.75 ± 8.14	19.33 (18.85, 21.19)	72.25 ± 4.59
*P*	0.390		0.062	0.063	0.057	0.342	0.644

**Table 2:** 24-Hour HRV indexes between the two groups.

Group	SDNN	RMSSD	SDANN	TP	LF	HF	LF/HF
Palpitations below the heart group	164.44 ± 31.48	42.38 ± 12.18	157.63 ± 35.88	2161.35 (1789.70, 2695.58)	571.25 (515.23, 689.20)	459.15 (232.98, 818.20)	1.46 (0.88, 1.73)
Normal group	157.38 ± 27.69	36.75 ± 7.38	137.00 (129.25, 162.25)	2337.91 ± 513.17	715.30 ± 241.20	384.84 ± 180.79	1.62 (1.48, 2.73)
*P*	0.596	0.245	0.462	0.624	0.426	0.462	0.159

**Table 3:** HRV indexes of the same group in different periods of day and night.

		Normal group		*P*	Palpitations below the heart group		*P*
		Day time	Nighttime		Day time	Nighttime	
Time domain indexes	SDNN	99.25 ± 19.54	148.13 ± 15.36	<0.001	103.50 (89.25, 114.50)	158.38 ± 46.10	0.009
	RMSSD	23.50 (22.00, 30.50)	49.25 ± 11.40	0.001	33.19 ± 8.18	54.81 ± 19.42	<0.001
	pNN50	4.00 (3.00, 9.50)	24.38 ± 9.18	0.001	11.63 ± 5.93	30.44 ± 14.17	<0.001

Frequency domain indexes	TP	1940.03 ± 411.77	2892.81 ± 798.83	0.004	1945.62 ± 406.98	2366.20 (1826.23, 3261.98)	0.006
	LF	622.01 ± 194.71	845.28 ± 326.74	0.012	548.48 ± 115.21	575.30 (431.90, 770.00)	0.163
	HF	147.85 (110.98, 209.18)	652.93 ± 327.21	0.004	221.85 (175.25, 408.78)	602.50 (364.30, 1465.45)	0.001
	LF/HF	3.87 ± 1.60	1.59 ± 0.93	0.002	2.38 ± 1.26	1.05 (0.62, 1.26)	0.005

The article "Correlation between Palpitations below the Heart in Traditional Chinese Medicine and Autonomic Nerve Function Based on Heart Rate Variability: A Case-Control Study" was published in 2021. Journal: Evid Based Complement Alternat Med.

**Table 4:** HRV indexes of different groups in different periods of day and night.

		Day time		*P*	Nighttime		*P*
		Normal group	Palpitations below the heart group		Normal group	Palpitations below the heart group	
Time domain indexes	SDNN	99.25 ± 19.54	103.50 (89.25, 114.50)	0.390	148.13 ± 15.36	158.38 ± 46.10	0.430
	RMSSD	23.50 (22.00, 30.50)	33.19 ± 8.18	0.042	49.25 ± 11.40	54.81 ± 19.42	0.465
	pNN50	4.00 (3.00, 9.50)	11.63 ± 5.93	0.027	24.38 ± 9.18	30.44 ± 14.17	0.286

Frequency domain indexes	TP	1940.03 ± 411.77	1945.62 ± 406.98	0.975	2892.81 ± 798.83	2366.20 (1826.23, 3261.98)	0.462
	LF	622.01 ± 194.71	548.48 ± 115.21	0.349	845.28 ± 326.74	575.30 (431.90, 770.00)	0.298
	HF	147.85 (110.98, 209.18)	221.85 (175.25, 408.78)	0.076	652.93 ± 327.21	602.50 (364.30, 1465.45)	0.806
	LF/HF	3.87 ± 1.60	2.38 ± 1.26	0.021	1.59 ± 0.93	1.05 (0.62, 1.26)	0.198

**Table 5:** Spearman correlation analysis of palpitations below the heart.

	Gender	Age	Abdominal circumference	Body mass index
Spearman correlation coefficient	0.389	0.237	−0.160	−0.198
*P*	0.061	0.266	0.454	0.354

**Table 6:** Spearman correlation analysis of palpitations below the heart.

	TP in daytime	LF in daytime	HF in daytime	LF/HF in daytime	SDNN in daytime	RMSSD in daytime	pNN50 in daytime
Spearman correlation coefficient	0.026	−0.115	0.370	−0.524	0.179	0.424	0.462
*P*	0.906	0.593	0.075	0.009	0.402	0.039	0.023

**Table 7:** Spearman correlation analysis of palpitations below the heart.

	TP in nighttime	LF in nighttime	HF in nighttime	LF/HF in nighttime	SDNN in nighttime	RMSSD in nighttime	pNN50 in nighttime
Spearman correlation coefficient	−0.153	−0.217	0.051	−0.268	0.096	0.121	0.147
*P*	0.475	0.308	0.813	0.205	0.656	0.572	0.493

**Table 8:** Logistic regression analysis of related factors of PBTH.

	*β*	Wald	OR	95% CI	*P*
RMSSD in daytime	—	—	—	—	0.771
pNN50 in daytime	—	—	—	—	0.851
LF/HF in daytime	−0.746	4.095	0.474	0.230–0.977	0.043

## Data Availability

All data included in this study are available upon request by contact with the corresponding author.
